RETRACTED

# Deep Learning Algorithm-Based Target Detection and Fine Localization of Technical Features in Basketball

**DOI:** 10.1155/2022/1681657

**Published:** 2022-05-23

**Authors:** WenHao Li, Yangyang Wu, BiZhen Lian, MingXin Zhang

**Affiliations:** ^1^China Basketball College, Beijing Sports University, Beijing 100084, Beijing, China; ^2^Tianfu College of Southwestern, University of Finance and Economics, Chengdu, Sichuan 610052, China; ^3^School of Physical Education and Training, Shanghai Institute of Physical Education, Shanghai 200438, Shanghai, China

## Abstract

Based on SSD to detect players, a super-pixel-based FCN-CNN player segmentation algorithm is proposed to filter out the complex background around players, which is more conducive to the subsequent pose estimation for target detection and fine localization of basketball technical features. The high resolution capability of CNN is used to extract images and perform computational preprocessing to identify typical basketball sports actions in video streams—rebounds, shots, and passes—with an accuracy rate of up to 95.6%. By comparing with three classical classification algorithms, the results prove that the target detection system proposed in this study is effective for target detection and fine localization of basketball sports technical features.

## 1. Introduction

Currently, Motion Capture System (MoCap) and related technologies have been widely used in the fields of sports science, biomechanics, and rehabilitation medicine [1, 2]. For example, the wearable Inertial Measurement Unit (IMU) contains components such as accelerometer, gyroscope, and magnetometer sensors, which can perform three-axis measurements and quantify acceleration, angular velocity, and direction of motion based on the hierarchical structure of human motion [3]. It has been successfully used for motion recognition in soccer, swimming, alpine skiing, and running due to its lightweight, wireless, and easy-to-use properties. However, in competitive competitions, the restricted experimental control conditions and the requirement to prohibit the affixing of marker dots and wearing sensors on the body surface suggest the disadvantages of the above motion capture techniques [4].

In recent years, markerless motion capture techniques based on computer vision have made human activity recognition in complex environments possible [5]. Through the camera equipment for markerless motion capture, the kinematic information in the game is obtained remotely, and the detected human activity is represented as wave signal features corresponding to specific actions and extracted to the computer terminal based on machine learning algorithm of computer vision, and then, the automatic analysis of video, automatic extraction of information, and fast feedback are completed simultaneously [6]. Action analysis based on computer vision images first needs to predict or estimate the position and direction of the target in the image sequence, by identifying targets with the same or similar features in consecutive images and then realizing real-time tracking and acquisition of displacement parameters. In current practical applications, the human body structure is usually reduced to a series of rigid bodies connected by frictionless rotating joints for easy identification and tracking by machines; however, in fact, the human body motion is very complex, and due to the muscle, tendon, and other factors, the human body motion is very complicated [7]. However, human motion is very complex and cannot be described by a simple rigid body model due to the presence of soft tissues such as muscles and tendons. Therefore, accurate tracking and quantification of dynamic human postures is one of the challenges faced by experts in computer vision, machine learning, and motion science [8].

RETRACTED

In addition, traditional machine learning algorithms have limited ability to process raw kinematic data, cannot effectively train on discontinuous, noisy, and high-dimensional data with missing values, and always require preprocessing of the original data, including Kalman Filter, Fast Fourier Transform, and Fourier Transform. The original data always need to be preprocessed, including Kalman Filter, Fast Fourier Transform (FFT), Master Fourier Transform (MFT), and dimensionality reduction including principal component analysis (PCA) and vector coding techniques [9]. It is noteworthy that the balance of robustness, accuracy, and effectiveness of computer-based motion analysis systems in competition sites depends on the improvement of algorithms and optimization of hardware compared to 3D motion capture analysis in laboratory environments. In recent years, automatic human pose recognition combined with deep learning (deep learning) algorithms has attracted extensive attention from experts and scholars in computer vision and other fields [10].

Deep learning is an important branch of machine learning characterized by a deeper neural network model architecture, the idea of which is derived from the biological neural network of the human brain [11]. Most of the algorithms use manually labeled image data to train neural networks and subsequently feed images or videos into the trained networks to perform estimation and recognition of human posture, joint centers, and bone positions [12, 13].

## 2. Related Work

In recent years, with the development of deep learning, some new solutions have emerged in the field of basketball video. The next section will introduce the deep learning methods in the field of basketball video. The first one is about the analysis of basketball and players and also plays in basketball videos, etc. A new recursive convolutional neural network for large-scale visual learning was developed in [14], which is not specific to basketball video analysis, but includes basketball videos in the dataset. Razakarivony and Jurie [15] analyzed a single-shot basketball game in life based on deep learning, and the method extracts spatial features of sampled frames as well as motion information in the video through VGG-16, followed by fusion of spatial and temporal features through a layer called ActionVLAD pooling, and the whole network is end-to-end structured. However, the basketball video analyzed in [16] is a one-person throwing scene and not a video of a multiplayer collaborative basketball game in an actual game. Zhengwan et al. [17] use deep learning to achieve basketball tracking, which is a method to determine whether a 3-point shot is successful by RNN, and the model can predict the trajectory of the basketball very well. An et al. [18] implement NBA tactical analysis based on deep learning, firstly, by locating the players as well as the relative position of the ball and, secondly, by implementing tactical classification based on convolutional networks. The latest literature [19] utilizes a two-way recurrent network BLSTM and a hybrid density network MDN framework to capture not only the basketball trajectory in real data but also the new trajectory of the sample. The application can automatically tell coaches and players when and where a shot is appropriate.

RETRACTED

Furthermore, regarding the analysis of basketball video events, the identification of multiplayer video events depends mainly on the performance of the participants and the interrelationships between the participants. Some studies have explored basketball events by studying the behavior of each participant and their relationships. Chandra et al. [20] proposed a model that combines detection and tracking of key players to achieve basketball event recognition, learning key players from all basketball players by applying the idea of attention mechanism, and finally combining information about other players and global information of video frames to achieve basketball event analysis, where information representation about players is achieved by CNN networks as well as BLSTM networks and representation about global information is the representation of global information achieved by CNN network and LSTM network. However, in the fast-motion team sports model, the extraction of key player regions tends to cause greater interference due to the existence of certain occlusions between players, and the algorithm has a complex framework and high computational complexity. It can be seen that the literature already has the ability to capture individual-level features, but the problem of player occlusion is very serious during basketball games, which tends to reduce the ability to track key players, and coupled with the complex background of basketball videos, this will lead to serious target confusion while the computational effort will increase dramatically.

RETRACTED

## 3. Research Methodology

International basketball tournaments or high-level basketball rivalry tournaments such as NBA usually have a relatively uniform shooting pattern system that can easily provide some image semantics of basketball events. According to the heterogeneous multiprocessor analysis method provided in the literature, this study is based on the analysis process of CNN heterogeneous multiprocessor basketball sports image detection, as shown in Figure 1, which uses the three most important actions in basketball: basketball standing, shooting, and passing to perform target detection and fine localization evaluation. Firstly, the convolutional neural network is applied to achieve frame-by-frame classification of basketball impact, keeping the structure and parameters of the layers before the fully connected layer of the existing convolutional neural network model unchanged, setting the number of nodes of the last fully connected layer to the number of image categories, and using migration learning to pretrain the parameters of the fully connected layer on Image Net to achieve end-to-end frame-by-frame image classification, whose network structure is shown in Figure 2, where the input of the CNN is an image frame and the output is a 4-dimensional vector:

(1) $$\begin{array}{c} O=\left[o_{1},o_{2},o_{3},o_{4}\right]. \end{array}$$

The assessment tasks for these three types of movements differ significantly from the current assessment algorithms for most movements, which are more fine arm movements, especially hand-basketball interactions, which are more skillful. Therefore, the existing movement evaluation methods are more difficult to be used to evaluate such fine movements. In order to fully exploit the activity dynamics of the human body during motion, edge noise reduction preprocessing of the image is required, when the original image is activated by an adaptive time-domain filter, which subtracts the blurred image from the original image and processes the image using the sharp edge formula to obtain a sharp image:

(2) $$\begin{array}{c} F\left(x,y\right)=2f\left(x,y\right)-f{}^{\prime }\left(x,y\right), \end{array}$$

where *f*(*x*, *y*) is the original image and *f*′(*x*, *y*) is the blurred image.

RETRACTED

Although time-domain filtering improves the accuracy of image sequence classification, a small number of misclassified image frames still exist, which may lead to finding the wrong boundaries. Therefore, in order to accurately extract advanced features for basketball action recognition associated with the video, the boundary localization algorithm improves the model to fit the video data and obtain higher accuracy [21].

There are 20 international top basketball players' game images in the image database, and each player's basketball action data contain about 18 000 images, and the size of each frame is adjusted to 64 × 48; then, the frames are input into the designed architecture for feature extraction. In order to train the parameters of the network, this study uses the stochastic gradient descent algorithm and sets the initial learning rate to 0.1, and after 10,000 iterations, the learning rate becomes 0.001 and sets the momentum to 0.9 and the weight decay to 0.000 2. This study trains the model until the training loss is overridden. Res Net-50 is chosen as the frame-by-frame image classification model for the CNN model, and all experiments are built on an Intel Xeon(R) with NVIDIA Quadro K5300 image processor, 32 GB RAM computer.

## 4. Results and Discussion

The results of the recognition and prediction of basketball players' movements by the target detection system in this study are shown in Table 1. The accuracy of prediction is the ratio of predicting a player's moving movements to the same value of ground truth. From Table 1, it can be seen that the accuracy of the recognition and prediction of the shooting motion of this method reaches more than 85%. However, the accuracy of rebound and pass recognition and prediction is low. The recognition accuracy and prediction accuracy on the test set are slightly lower than those on the valid set, which indicates that the performance of the target detection system model in this study can be further improved by more significant training examples [22, 23].

For a specific basketball game, the target detection system is reconstructed based on the key points of the human body for the corresponding actions, basketball, shooting, and passing. The method proposed in this study can help basketball players to adapt to various training methods and tactics to a certain extent and improve their performance quickly. A linear regression analysis was conducted to investigate the correlation between the automatic scoring of the target detection system (the algorithm proposed in this study) and the traditional manual scoring in rebounding, shooting, passing, and fine motor assessment, respectively, as shown in Figure 3(a). Each point in Figure 3(b) represents the result of one test, the horizontal coordinate indicates the assessment score obtained by the automatic assessment algorithm, and the vertical coordinate indicates the true value assessed by the traditional training method. From Figure 3(c), it can be seen that the automatic assessment algorithm and the traditional training method scores are linearly related. Compared with the traditional training methods, the fine movements obtained by the target detection system in this study (Figure 3(d)) have certain advantages and can bring better teaching effects. This combination of explanation and demonstration can greatly stimulate the athletes' senses and lead to a deeper memory and understanding of the technique [24].

RETRACTED

In addition, traditional models generally fail to recover some arm posture characteristics of basketball, such as severe blocking, high movement speed, sudden directional changes, and a large number of physical confrontations between players, which challenge the accuracy of detection efficiency of individual players and teams. Therefore, the target detection and fine localization method proposed in this study obtains a more refined detection and fine localization method by cropping the area where the detected player is located after the detection of the player and dividing five motion channels to characterize the arm pose distribution by the statistics of the arm pose features to identify the affiliation of the basketball playing style. Since the a priori condition of uniform arm posture is obtained, this method can classify the basketball hitting affiliation without additional annotation during the construction of the dataset and can identify the technical skills of basketball far mobilization more accurately. With integral channel features (ICF) [11], fast recursive results are similar to those of ICF [11], Faster Recurrent Convolution Neural Network (RCNN), Single Shot Multibox Detector (SBMD), and the Faster RCNN [25, 26].

The results are shown in Figure 4. It can be seen that this method has the highest accuracy among all the algorithms, reaching 95.6%, which indicates that the target detection system designed in this study is effective [27].

To demonstrate the effectiveness of GCMPs, this experiment implements the classification of 5 types of events (3-pointers, free throws, layups + other 2-pointers, dunks, and steals) in 2 ways according to the framework in Figure 5. One way is the complete framework of Figure 5, and the other way is to disregard the GCMPs part in Figure 5 and directly input the original video frames to the CNN network to achieve feature extraction. The comparison results are shown in Table 2.

RETRACTED

From Table 2, we can see that the accuracy of free throw, layup + other 2-pointers, dunk, and steal classification increased by 72.13%, 12.76%, 10.83%, and 27.36%, respectively, after adding GCMPs, while the accuracy of 3-pointers only decreased by 0.76%. The average accuracy can be improved by 18.46%. Therefore, we believe that GCMPs are effective for event classification.

The analysis shows that the event-occ video segment has less event correlation except for the layup and the other 2-pointers. To verify this, we extract GCMP_DF_SVF features from the event-occ video segment to achieve the 6 classification of events. The confusion matrix of the classification results is shown in Table 3.

As shown in Table 3, the average prediction accuracy is 58.22%, in which the classification accuracy of 3-pointers, free throws, and steals events can reach more than 60%, but only about 20% for layups and dunks. From row 4 of the table, it can be found that 35% of the layup video segments are misclassified as other 2-pointers. It can be seen that the results of the 2-stage classification algorithm improve the classification accuracy of the layup and other 2-point events by 21.26% and 6.41%, respectively. The other events also changed by +5.12%, −2.55%, −3.22%, and −10.56%, respectively, but the average result improved by 2.74%. This result proves that our proposed 2-stage event classification method based on event-occ is effective.

## 5. Conclusion

Computer vision-based markerless motion captures basketball sports application in the areas of motion technique recognition and sports performance analysis in this study. We design the development and application of deep learning algorithms such as CNN and RNN, which are better than traditional machine learning methods for motion capture and recognition in some scenarios.

Future research can compare traditional machine learning algorithms with deep learning recognition algorithms for specific motion action recognition and motion performance evaluation, so as to provide a basis for the selection and fusion application of motion recognition techniques and related algorithms. Computer vision images can be used in conjunction with wearable wireless inertial sensing and other devices to achieve joint multiparameter acquisition of motion processes and improve the effectiveness, efficiency, and robustness of markerless action recognition.

## Figures and Tables

**Figure 1:** CNN fine-motion evaluation process.

RETRACTED

**Figure 2:** Schematic diagram of CNN structure for image classification.

**Figure 3:** Correlation analysis between automatic scoring of target detection system and traditional manual scoring. (a) Rebounding; (b) shooting; (c) passing; (d) fine motor.

**Figure 4:** Comparison of the method in this study with other methods.

**Figure 5:** An overview of GCMP-based event recognition.

**Table 1:** Comparison of recognition results and prediction results of basketball players' movements.

Action classification	Effective accuracy		Test training accuracy	
	Recognition result (%)	Forecast result (%)	Recognition result (%)	Forecast result (%)
Rebounding	88	86	84	83
Shooting	92	91	87	84
Passing	93	90	82	81

**Table 2:** Comparison of event classification performance with/without GCMPs on event-occ segments.

Accuracy (%)	No GCMPS	With GCMPS
3-Pointer	69.32	68.56
Free throw	20.86	92.99
Layup + other 2 points	72.22	74.98
Filling ball	5.36	16.13
Snatch	80.21	68.11
Average accuracy (%)	49.65	68.11

**Table 3:** Confusion matrix for GCMP_DF_SVF-based event classification on event-occ segments.

Forecast/label	3-Pointer	Free throw	Layup	Other 2 points	Filling ball	Snatch	Accuracy (%)
3-Pointer	347	12	9	118	7	54	63.44
Free throw	4	150	0	0	0	3	95.54
Layup	44	12	98	153	25	96	22.90
Other 2 points	127	28	50	333	12	121	49.63
Filling ball	18	2	0	1	6	4	19.35
Snatch	1	4	0	2	0	438	98.43
Average accuracy (%)	...	...	...	...	...	...	58.22

## Data Availability

The raw data used to support the findings of the study can be obtained from the corresponding author upon request.
